The article "The Potential Role of Gut Peptide Hormones in Autism Spectrum Disorder" was published in 2020. Journal: Front Cell Neurosci.

# The Potential Role of Gut Peptide Hormones in Autism Spectrum Disorder

**DOI:** 10.3389/fncel.2020.00073

**Published:** 2020-03-31

**Authors:** Xin-Rui Qi, Li Zhang

**Affiliations:** ^1^Center for Translational Neurodegeneration and Regenerative Therapy, Shanghai Tenth People’s Hospital Affiliated to Tongji University School of Medicine, Shanghai, China; ^2^Joint International Research Laboratory of CNS Regeneration, Guangdong-Hong Kong-Macau Institute of CNS Regeneration, Jinan University, Guangzhou, China

**Keywords:** autism, cholecystokinin, ghrelin, gut peptide hormone, pituitary adenylate cyclase activating peptide, secretin, vasoactive intestinal peptide

## Abstract

Gut peptide hormones are one group of secretory factors produced from gastrointestinal endocrine cells with potent functions in modulating digestive functions. In recent decades, they have been found across different brain regions, many of which are involved in autism-related social, emotional and cognitive deficits. Clinical studies have revealed possible correlation between those hormones and autism spectrum disorder pathogenesis. In animal models, gut peptide hormones modulate neurodevelopment, synaptic transmission and neural plasticity, explaining their behavioral relevance. This review article will summarize major findings from both clinical and basic research showing the role of gut peptide hormones in mediating autism-related neurological functions, and their potential implications in autism pathogenesis. The pharmaceutical value of gut hormones in alleviating autism-associated behavioral syndromes will be discussed to provide new insights for future drug development.

## Introduction

Autism spectrum disorder (ASD) affects more than 1.5% of children worldwide (Christensen et al., 2016). It is estimated that genetic factors contribute to about 60% of ASD cases (Tick et al., 2016) although there are still episodic cases that cannot be fully explained by hereditary factors. Emerging evidence is suggesting gut dysfunctions in ASD, which is frequently correlated with digestive disorders. Typical gastrointestinal (GI) symptoms associated with ASD include abdominal pain, flatulence, indigestion or diarrhea (Adams et al., 2011), whose incidence were as higher as 70% in ASD children (Li and Zhou, 2016).

Gut peptide hormones refer to a group of polypeptides derived from GI tract and can exert multiple physiological functions via binding with specific receptors. Gut peptides have a long history since the identification of its first member, secretin, at almost 100 years ago. Currently dozens of molecules have been classified into this group, including cholecystokinin (CCK), vasoactive intestinal peptide (VIP), pituitary adenylate cyclase activating peptide (PACAP), peptide YY (PYY), secretin, pancreatic polypeptide, ghrelin and so on (Small and Bloom, 2004; Wren and Bloom, 2007; Neary and Batterham, 2009). Those secretory factors have been recognized for their roles in modulating GI functions and body energy metabolism. In recent 20∼30 years, their brain functions are being gradually revealed from molecular, behavioral and physiological evidence (Zhang and Chow, 2014; Donahue et al., 2016; Kingsbury and Wilson, 2016). For example, CCK and VIP are now working as markers for specific sub-population of neurons having unique morphological features of axon collaterals and firing patterns (Kawaguchi and Kondo, 2002). On the other hand, gut peptides also directly participate in the regulation of neural functions across different brain regions. Among those neurological effects, people are more familiar with the central appetite control in which gut peptides can sense the satiety and energy requirement, and mediate the activity of central feeding nuclei within arcuate nucleus (Arc) of the hypothalamus and the nucleus of the solitary tract (NTS) via vagal afferent pathway or direct effects on central nuclei (Konturek et al., 2004; Small and Bloom, 2004; Wren and Bloom, 2007; Troke et al., 2014; Roman et al., 2017).

The article "The Potential Role of Gut Peptide Hormones in Autism Spectrum Disorder" was published in 2020. Journal: Front Cell Neurosci.

Besides the feeding and metabolic regulation, the potential role of gut peptide hormones in other behavioral paradigms is emerging in recent decades. Notably, some gut peptides are involved in social functions. Examples include secretin, whose gene knockout in mice leads to social interaction deficits (Nishijima et al., 2006), and VIP with potent functions for social affiliation and aggression (Kingsbury and Wilson, 2016). As social deficit is one of core symptoms of ASD, one may speculate that gut peptides are related with ASD pathogenesis. Therefore, further understandings of gut peptide hormones in ASD should help to better elucidate both pathogenic mechanism and to develop potential intervention strategy of ASD.

In this mini review, for each gut peptide hormone we will start with its distribution and functions in the central nervous system, following with the evidence of its involvement in ASD. We will also discuss about the neurobiological mechanisms of those gut-brain peptides, with particular interests in mediating social and cognitive deficits as well as stereotypic behaviors, all of which are the core behavioral symptoms of ASD. Lastly, the potency of drug development targeting those gut peptides and their receptors in alleviating ASD-related symptoms will be discussed.

## Gut Peptide Hormones and ASD

Gut peptide hormones exert various neuromodulating effects as suggested by their wide distribution across different brain regions. Recent advances in neural science techniques including gene knockdown, *in vivo* recording, opto-/chemo-genetics have made it possible to delineate specific functions of those peptides within certain neural circuits including those related with ASD.

The article "The Potential Role of Gut Peptide Hormones in Autism Spectrum Disorder" was published in 2020. Journal: Front Cell Neurosci.

### CCK

As one widely studied gut-brain peptide, CCK can be found within a certain group of inhibitory neurons and has known effects in mediating appetite and food intake (Degen et al., 2001). Previous studies have found that social isolation increases CCK mRNA expression in amygdala, hippocampus, cortex and ventral tegmental area (VTA) nuclei of rats (Del Bel and Guimaraes, 1997). Clinical assays also showed that decreased serum CCK-8 (Brambilla et al., 1997) is found in ASD children. Furthermore, in patients with Asperger’s syndrome (AS), a subgroup of autistic patients, one fragment deletion has been found in CCK gene (Iourov et al., 2015). Those animal and clinical data thus suggest the possible linkage between CCK and ASD.

Some studies have already been done to investigate the potential neurological mechanisms of CCK in social behaviors. Targeted mutation of CCK receptor alters social isolation-related behaviors in female mice (Abramov et al., 2004). The selective activation of CCK-neurons (Whissell et al., 2019) and selective modulation of CCK receptors (Lemaire et al., 1992) enhances social recognition or social memory. At the upstream of CCK, endocannabinoid system plays a critical role. In hippocampal nuclei, endogenous cannabinoid receptor 1 (CB1R) suppresses CCK-positive neurons, leading to altered social behaviors (Vargish et al., 2017). Further analysis showed that CB1 modulated CCK transmission to direct social withdraw behaviors (Seillier et al., 2013). A recent study also found that CB1R in the amygdala CCK-positive afferents to nucleus accumbens modulates social defeat-induced depressive behaviors (Shen et al., 2019). The inter-correlation between endocannabinoid and CCK system may reside in the co-expression of CB1R and CCK in certain groups of interneurons (Rovira-Esteban et al., 2017). In future, more studies can be performed to elucidate the neural circuit of CCK in mediating social behaviors.

### PACAP

PACAP is one polypeptide hormone sharing high sequence similarity with secretin and is also involved in social modulation. Genetic study investigated more than 1,000 ASD children with their normal siblings and identified one specific loci (rs1557299) at the downstream of PACAP gene (Nijmeijer et al., 2010) which suggested close relationship between PACAP and ASD. Furthermore, animal studies showed that PACAP is an important gut peptide in modulating social and emotional behaviors. For example, the intracerebroventricular infusion of PACAP into rat brains leads to the decrease of social behaviors (Donahue et al., 2016). On the other hand, PACAP – deficient mice presented the attenuation of depressive disorders after chronic social defeat stress (Lehmann et al., 2013). However, the knockout of PACAP type 1 receptor (PAC1) in male mice decreased social investigations after repeated exposure to the same subject, in conjunction with excessive sexual mounting and lower aggressive behaviors (Nicot et al., 2004). Those seemingly contradictory phenotypes suggest the homeostatic regulation of PACAP in maintaining normal social behaviors. The administration of PACAP also leads to prominently enhanced locomotor activity plus rearing behaviors in mice (Masuo et al., 1995; Norrholm et al., 2005), and the deficiency of PACAP in mice results in hyperactivity and jumping behaviors in a novel field (Hashimoto et al., 2001). Therefore, PACAP mediates various behavioral phenotypes that can be related with ASD.

The article "The Potential Role of Gut Peptide Hormones in Autism Spectrum Disorder" was published in 2020. Journal: Front Cell Neurosci.

Electrophysiological studies reveal that PACAP improves synaptic plasticity in mouse hippocampus (Cabezas-Llobet et al., 2018), and increases both frequency and amplitude of excitatory postsynaptic currents (EPSCs) of autonomic synapse (Starr and Margiotta, 2017), giving clues of how PACAP is involved in the autism-related behaviors. In addition, studies are gradually revealing the modulatory function of PACAP in neurodevelopment and neuroprotection, which might give further explanation for its involvement in ASD, which is one neurodevelopmental disorder. As further evidence, PACAP can stimulate the growth of both axons (Ogata et al., 2015) and dendritic spines (Cabezas-Llobet et al., 2018) under normal or disease conditions. Moreover, PACAP receptor PAC1 also mediates the differentiation and migration of cortical neuronal progenitors (Adnani et al., 2015).

### VIP

VIP is mainly expressed in the hypothalamic nuclei such as suprachiasmatic nucleus (SCN) and tuberal hypothalamus as well as hippocampus and cerebral cortex (Acsady et al., 1996a, b), and is now commonly accepted as a neuroendocrine hormone, putative neurotransmitter and cytokine. Its biological effects are mediated by binding to the G-protein coupled receptors (GPCRs), VPAC1 and VPAC2, which have high affinity to VIP (Iourov et al., 2015). Previously, it has been shown to stimulate prolactin secretion from the pituitary (Reichlin, 1988) and catecholamine release from the adrenal medulla (Malhotra et al., 1988). It also participates in non-adrenergic, non-cholinergic relaxation of both vascular and non-vascular smooth muscle as co-transmitters with nitric oxide and carbon monoxide (Said and Rattan, 2004).

The article "The Potential Role of Gut Peptide Hormones in Autism Spectrum Disorder" was published in 2020. Journal: Front Cell Neurosci.

Recent evidence suggested a close relationship between VIP and ASD. Newborns with higher VIP concentrations in the cord blood were more likely to develop autism in later periods (Nelson et al., 2001). Preliminary evidence has showed that ASD phenotype is associated with VPAC2 receptor duplication (Levinson et al., 2011). The involvement of this duplication in ASD is further confirmed by a recent report observing such copy number variants in autistic child and his father with a mild autism (Firouzabadi et al., 2017). Preclinical studies support the roles of VIP in social and cognitive functions. After VIP antagonist treatment during the embryonic stage, male offspring exhibited reduced sociability and deficits in cognitive function, as assessed through cued and contextual fear conditioning (Hill et al., 2007). Male offspring of pregnant females with VIP deficiency also exhibited deficits in social approach behavior and reversal learning, with more severe and higher prevalence compared to their female littermates (Lim et al., 2008; Stack et al., 2008). VIP-deficient mice exhibited a pronounced reduction in social recall when tested 48-h or longer after primary training (Chaudhury et al., 2008). On the other hand, some early studies showed that the intracerebroventricular administration of VIP also caused a marked impairment in passive avoidance and spatial memory, together with neuronal dystrophy (Takashima et al., 1993a, b). As further supporting evidence, VIP can stimulate neurogenesis as well as cell differentiation to promote neuronal survival and regeneration probably via the induction of nerve growth factor and activity dependent neuroprotective protein (Hill et al., 2002; Giladi et al., 2007). In addition, VIP has been observed to modulate synaptic transmission efficiency via the regulation of brain-derived neurotrophic factor (BDNF) expression in cortical neurons (Pellegri et al., 1998; Ciranna and Cavallaro, 2003), providing possible mechanism for behavioral modulation.

### Ghrelin

Ghrelin, a 28-amino-acid peptide hormone, is mainly produced by gastric oxyntic cells. In the central nervous system, ghrelin has been detected in the hypothalamus such as Arc, ventromedial and paraventricular nucleus areas (PVN) (Kojima et al., 1999; Lu et al., 2002; Hori et al., 2008). The hypothalamic roles of ghrelin consist of appetited regulation, glucose homeostasis, and growth hormone release from pituitary and body weight regulation (Kojima and Kangawa, 2005). Furthermore, ghrelin is found in extra-hypothalamic areas such as hippocampus, sensory-motor cortex and cingulate cortex which might be involved in higher cognitive functions (Hou et al., 2006). Ghrelin is present in two major forms: un-acylated ghrelin (des-acyl ghrelin or DAG) and acylated ghrelin (AG, C-ghrelin, or also referred to as ghrelin) which was produced by ghrelin *O*-a-cyl-transferase (GOAT) from DAG. Only AG is able to bind to the growth hormone secretagogue receptor type 1 a (GHSR1a), a G protein-coupled receptor, to execute their biological functions (Kojima et al., 1999, 2001). GHSR1a is widely distributed in the brain such as in the hypothalamus, hippocampus, substantia nigra, VTA and several thalamic and brain stem nuclei (Guan et al., 1997). Those expressional data indicate the potential neural function of ghrelin.

The article "The Potential Role of Gut Peptide Hormones in Autism Spectrum Disorder" was published in 2020. Journal: Front Cell Neurosci.

Recent study revealed the close relationship between ghrelin and ASD. For example, the expression level of un-acylated ghrelin acylated ghrelin in blood is lower in children with autism (Al-Zaid et al., 2014). Ghrelin has also been postulated to be one promising target in co-morbid between autism and epilepsy (Ghanizadeh, 2011). Animal studies show that ghrelin plays important roles in learning and memory, sleep and appetite, all of which are disturbed in ASD. Intracerebroventricular or intra-hippocampal injection of ghrelin increased memory acquisition and/or consolidation, but not in memory retrieval (Carlini et al., 2002, 2010). Ghrelin-knockout mice exhibited decreased hippocampal spine density and abnormal memory that can be reversed by ghrelin injection (Diano et al., 2006). In addition, GHSR1a knockout mice showed a decreased food intake after three days on restricted feeding schedule and failed to show preference to rewarding high-fat diet food (Abizaid et al., 2006), suggesting the role of ghrelin in reward circuitry modulation. In physiological terms, ghrelin was found to enhance synaptic plasticity by increasing spine formation and long term potentiation (LTP), to promote neurogenesis (Zhang et al., 2004; Moon et al., 2009), to preserve mitochondrial integrity, and to inhibit the apoptotic process and neuronal cell death (Chung et al., 2007; Lee et al., 2010). Moreover, ghrelin was recently reported to reduce mRNA expression of tumor necrosis factor-α (TNF-α) and nuclear factor kappa B (NF-κB) in lymphoblastoid cell lines from ASD subjects (Yamashita et al., 2019), suggesting the possible involvement of neuroinflammatory modulation of ghrelin.

### Secretin

Secretin is one classical gut-peptide hormone to modulate pancreatic secretion as well as body energy homeostasis. Several lines of evidence from rodent and human studies show that secretin and its receptors are widely distributed in the brain areas from cerebral cortex, hippocampus, amygdala, hypothalamus to cerebellum (Yuan et al., 2011; Wang et al., 2019). The neurological functions of secretin are also being gradually explored by molecular, physiological and behavioral approaches (Zhang and Chow, 2014; Wang et al., 2019).

The article "The Potential Role of Gut Peptide Hormones in Autism Spectrum Disorder" was published in 2020. Journal: Front Cell Neurosci.

In 1998, a case series reported secretin in amelioration of the symptoms in three ASD children (Horvath et al., 1998). However, later double-blind placebo-controlled clinical studies revealed that there was a lack of significant impact of secretin in the treatment of ASD symptoms (Esch and Carr, 2004; Malone et al., 2005; Krishnaswami et al., 2011; Lyra et al., 2017). In spite of the failure in clinical studies, animal obervations support the roles of secretin in some social functions. For example, secretin receptor deficient mice presented impaired social interaction (Nishijima et al., 2006), and one later study revealed the potentiation of social recognition by secretin infusion via the activation of oxytocin pathway (Takayanagi et al., 2017). One possible mechanism exists as secretin increases the release of vasopressin (Chu et al., 2009) which can regulate social behaviors (Dumais and Veenema, 2016). Besides social regulation, in a mutant mouse model with stereotypically circling locomotion, secretin infusion effectively attenuated those abnormalities (Koves et al., 2011). Altogether, these data might indicate an indirect roles played by secretin in the ASD pathogenesis and treatment.

For investigating the molecular and cellular mechanism, secretin has been found to induce the spinogenesis of hippocampal neurons (Nishijima et al., 2006), and the deficiency of secretin impairs both the induction and maintenance of LTP in hippocampal neurons (Yamagata et al., 2008). We recently found that secretin could potentiate postnatal proliferation and migration of cerebellar granular neurons (Wang et al., 2017) and potentiate inhibitory postsynaptic currents (IPSCs) of cerebellar Purkinje neurons (Yung et al., 2001), adding further knowledge to the neural plasticity modulation by secretin. As the secretin receptors mostly belong to GPCR family, the activation of cyclic AMP (cAMP)–protein kinase A (PKA) pathway in brain regions have been established for secretin (Pang et al., 2015). This also holds true for VIP and PACAP, which have high degree of sequence similarity with secretin (Jozwiak-Bebenista et al., 2015). The activation of cAMP–PKA pathway exerts pluripotent functions, among which the modulation of ion channels or neurotransmitters directly affects synaptic transmission (Wang et al., 2019). Alternatively, other downstream pathways such as cAMP-response element – binding protein (CREB) activation (Mak et al., 2019) can initiate the translation of synaptic proteins to modulate long-term plasticity and memory functions. The extracellular signal regulated kinase (ERK) pathway is also involved upon secretin stimulation (Wang et al., 2017). In sum, secretin is one possible modulator of social functions, and is worth further investigation to reveal detailed circuitry effects.

The article "The Potential Role of Gut Peptide Hormones in Autism Spectrum Disorder" was published in 2020. Journal: Front Cell Neurosci.

## Implications for Autism Drug Development

Based on the inter-correlation between ASD pathogenesis and potentially neurological mechanisms in regulating social, emotional and repetitive behaviors by gut peptides, it is expected that those hormones may work as drug candidate or targets for developing novel drugs in alleviating ASD symptoms. However, failures are frequently reported when directly trying the administration of those peptides to ameliorate autistic behaviors. For example, one clinical trial failed to detect significantly improvement of social phobia by using CCK-tetrapeptide (CCK-4) (Katzman et al., 2004), and many double-blind placebo-controlled studies using secretin to alleviate autism symptoms infusion have also been failed (Esch and Carr, 2004; Malone et al., 2005; Krishnaswami et al., 2011; Lyra et al., 2017) even though the existence of one early study reporting the beneficial effects of secretin (Horvath et al., 1998). Therefore, major challenges are faced by those gut hormones probably due to their rapid turnover *in vivo* and low efficiency for penetrating the blood brain barrier (BBB). Large amounts of works are thus required to overcome those disadvantages and to generate drug candidates with satisfactory efficiency, persistency and safety.

The short half-life is one common property of gut hormones due to their peptide composition. For example, secretin has less than 5 min half-life under normal physiological conditions (Kolts and McGuigan, 1977), making it impossible to achieve stable drug concentration *in vivo*. Such limitation can be addressed by two approaches: the development of stable analog or receptor agonist, or the application of bioengineered sustained drug delivery system. The former approach is based on molecular design and screening of small molecules, or the modification of existing receptor ligands, to generate long-lasting effects as those of natural ligands. Alternatively, one can adopt nanoparticles system to chronically release peptide drugs such as those used in immunomodulation therapy for releasing autoantigens (Stabler et al., 2019). In drug development, the issue of BBB permeability should also be considered case-by-case. Current knowledge agree that VIP, secretin and PACAP27 can be transported into the brain by a non-saturable mechanism, or transmembrane diffusion, whilst PACAP38 and gastric inhibitory polypeptide (GIP) have no known routes in enter the central nervous system (Dogrukol-Ak et al., 2004). Those data thus suggest that it is necessary to develop new drug delivery system to penetrate the BBB and to chronically release effective gut peptide hormones.

The article "The Potential Role of Gut Peptide Hormones in Autism Spectrum Disorder" was published in 2020. Journal: Front Cell Neurosci.

## Conclusion

Gut peptide hormones are now recognized as having prominent brain distributions and various behavioral modulatory functions. Clinical studies with ASD subjects have revealed that the genetic polymorphisms of gut peptides such as CCK, PACAP, and VIP are related to ASD. Altered expression levels of the peptides including CCK and ghrelin are found in ASD children. Additionally, more animal studies suggest that these gut peptides are actively involved in the modulation of social, emotional and stereotypic behaviors. In future, one should perform more site-specific studies to illustrate the precise mechanisms of gut peptides in mediating social or emotional or cognitive behaviors for potential drug targets. Further drug development can be pursued to generate stable analogs that can modulate gut peptide pathways in the brain, aiming to relieve behavioral symptoms of ASD.

## Author Contributions

X-RQ wrote the manuscript with the help from LZ. LZ revised the manuscript.

## Conflict of Interest

The authors declare that the research was conducted in the absence of any commercial or financial relationships that could be construed as a potential conflict of interest.
